# Clinically Healthy Human Gingival Tissues Show Significant Inter-individual Variability in GCF Chemokine Expression and Subgingival Plaque Microbial Composition

**DOI:** 10.3389/froh.2021.689475

**Published:** 2021-07-14

**Authors:** Shatha Bamashmous, Georgios A. Kotsakis, Sumita Jain, Ana M. Chang, Jeffrey S. McLean, Richard P. Darveau

**Affiliations:** ^1^Department of Periodontics, University of Washington, Seattle, WA, United States; ^2^Department of Oral Health Sciences, University of Washington, Seattle, WA, United States; ^3^Department of Periodontology, Faculty of Dentistry, King Abdulaziz University, Jeddah, Saudi Arabia; ^4^Department of Periodontics, University of Texas Health Science Center, San Antonio, TX, United States; ^5^Department of Microbiology, University of Washington, Seattle, WA, United States

**Keywords:** gingiva, gingival crevicular fluid, chemokine, gingival health, subgingival microbiome, host response

## Abstract

**Aim:** Clinically healthy gingival tissue is maintained through controlled regulation of host defense mechanisms against plaque biofilm overgrowth. One key component is the transit of neutrophils from the vasculature into gingival tissue where the expression of different neutrophil chemokines are tightly regulated. This cross-sectional study examines the inter-individual variability in chemokine profiles within gingival crevicular fluid (GCF) in relation to the subgingival bacterial community in a state of gingival health.

**Methods:** Gingival crevicular fluid and subgingival plaque samples were collected from mesiobuccal surfaces of all six Ramfjord teeth of 20 systemically healthy individuals (14.55 ± 1.67 years). A multiplex immunoassay was carried out to quantify the expression of 40 different chemokines in the healthy gingival tissue. Neutrophils were assessed indirectly by myeloperoxidase (MPO) in GCF using traditional ELISA. Characterization of healthy subgingival plaque was conducted with the Illumina Miseq targeting the 16S rRNA gene.

**Results:** In health, there are distinct variations within individual gingival crevicular fluid chemokine expression profiles, as well as in the concentration of neutrophils, that divided the participants into high or low chemokine expressing groups. Specifically, key differences were identified within MIF (2683.54 ± 985.82 pg per 30-s sample), IL-8/CXCL8 (170.98 ± 176.96 pg per 30-s sample), Gro-α/CXCL1 (160.42 ± 94.21 pg per 30-s sample), ENA-78/CXCL5 (137.76 ± 76.02 pg per 30-s sample), IL-1β (51.39 ± 37.23 pg per 30-s sample), TNF-α (1.76 ± 1.79 pg per 30-s sample), and IFN-γ (0.92 ± 0.54 pg per 30-s sample). Of these identified chemokines, the highest correlation was associated between IL-8/CXCL8 and neutrophils (*r* = 0.54, *p* = 0.014). Furthermore, species characterization of healthy subgingival plaque revealed significant inter-individual variability that identified two unique groups unrelated to the previously identified chemokine groups.

**Conclusion:** The lack of concordance between the microbial composition and chemokine profile during health may be a reflection of the unique microbial composition of each individual coupled with variations within their host response, emphasizing the vast complexity of the defense mechanisms in place to maintain gingival health.

## Introduction

Neutrophils are a crucial component of periodontal health representing the first line of defense against microbial challenge [1]. The migration and activation of these key effector cells within the gingiva are orchestrated by complex networks of host mediators called chemokines and cytokines. Studies have shown that bacteria have an influential role in the immunomodulation of host mediators and hence, the host response. It has been demonstrated that neutrophil homing to clinically healthy tissue, similar to the inflammatory response, is a highly selective process where the expression of different neutrophil chemoattractants, such as CXCL1, CXCL2, and CXCL6 are regulated both spatially and temporally in response to oral commensal bacteria colonization in the mouse [2, 3]. Similarly, humans are highly selective in the expression of neutrophil chemokines in both periodontal health and disease [4, 5]. Thus, the crucial role of neutrophils in periodontal homeostasis is of great interest; in particular, the role of chemokine expression within each stage of periodontal pathogenesis. However, since most studies have zeroed into the passive understanding of health through direct comparisons to disease, little is known about the proactive roles of the host response during the maintenance of periodontal health.

The chemokines' role in the amplification of the host immune response can be linked to the pathogenesis of various inflammatory diseases. Indeed, dysregulation of the host immune response, as well as the dysbiosis of the oral microbial community, have been attributed to the pathogenesis of periodontal disease [6]. For example, a study using the CRISPR/Cas9 system to engineer and test previously identified human haplotypes within the interleukin-8 gene (IL-8; also known as CXCL8) have provided new evidence of the active involvement of host genetics to increase neutrophil migration *in vitro* and hence its potential to influence an individual's susceptibility to disease [7]. Furthermore, there is growing awareness behind the host protective role of the microbial dental plaque biofilm as a key player for the maintenance of healthy homeostasis [8, 9]. Studies by To et al. and Myers et al. have shown the unique immunosuppressive potential of healthy subgingival and supra-gingival plaque, respectively [10, 11]. However, limited investigation into these interactions between the subgingival microbial community and the host immune response have provided insufficient information to detangle this relationship [12, 13]. Nevertheless, a complete understanding of the contributions of the various microbial communities in association with the innate host immune response during health or disease is essential for the field. Therefore, a full assessment of the host-bacterial interaction in health is necessary to further our understanding of the etiology of periodontal disease and identify novel biomarkers of this disease.

This study more broadly characterized the subgingival microbiome and the host immune response in gingival health. A comprehensive evaluation of 40 major inflammatory mediators within the gingival crevicular fluid (GCF) of 20 healthy subjects revealed that the healthy host inflammatory response is a highly variable and dynamic process that does not seem to show direct association with the oral microbial composition. Altogether, this data demonstrates the highly complex and dynamic nature of health that is unique for each individual in regards to both the host response and microbiome; and hence suggests that there may not be a single defined path to periodontal health.

## Materials and Methods

### Study Population

As a pilot exploratory study performed for feasibility, power analysis was not performed. The selection of 20 participants for this study was chosen for convenience.

This study was approved by the University of Washington Human Subjects Review Committee (HSD#46857). Following the principles of the Declaration of Helsinki, 20 systematically healthy adolescents aged 12–17 were enrolled after undergoing parental consent and individual assent. In order to limit hormonal influences on this data set, this study utilized strict entry criteria. For eligibility, subjects had gingival health with no clinical signs of gingival inflammation at the time of screening using diagnostic criteria from the 2017 World Workshop Classification [14]. Exclusion criteria included: antibiotic therapy or anti-inflammatory drugs within 90 days of enrollment, and history of smoking and periodontal disease.

### Clinical Data and Biospecimen Collection

After enrollment, participants underwent an additional abbreviated periodontal health assessment on the Ramfjord teeth to ensure gingival index (GI) = 0, probing depth (PD) ≤ 3.0 mm, absence of bleeding on probing (BOP), and absence of attachment loss for the study teeth. Ramfjord teeth include specific sites that are consistently used for periodontal clinical research studies including upper right 1st molar, upper left central incisor, upper left 1st premolar, lower left 2nd molar, lower right central incisor, and lower right 1st premolar [15]. All clinical measurements, including probing depth (PD), visible plaque index (VPI) [16], gingival index (GI) [17], and bleeding on probing (BOP) were performed by a single, trained examiner S.B. using a periodontal probe (UNC-15, Hu-Friedy, Chicago, IL, USA). All measurements were assessed at six surfaces per tooth: mesiobuccal, direct buccal, distobuccal, distolingual, direct lingual, and mesiolingual. The BOP was recorded within 20 seconds of probing.

Immediately following clinical examination, collection of gingival crevicular fluid (GCF) and subgingival plaque samples were performed within the same visit. Both plaque and GCF samples were collected from the mesiobuccal surfaces of Ramfjord teeth [15], which were isolated with cotton rolls and gently air-dried. GCF samples were collected first with sterile paper strips (Periopaper; Oraflow Inc., Smithtown, NY, USA) that were inserted into the gingival crevice until mild resistance was felt and left in place for 30 seconds. The volume of GCF was measured with a calibrated measuring device (Periotron 6000; Oraflow Inc., Smithtown, NY, USA) and converted into fluid volume (μl) using the provided software (Periotron Professional 3.0 software; Oraflow Inc., Smithtown, NY, USA) [18]. GCF samples were collected from the mesiobuccal surfaces of all six Ramfjord teeth and pooled into a single 1.5 ml microcentrifuge tube. After collection, GCF samples were stored immediately on ice and transported to the lab for processing.

Similarly, subgingival plaque samples were collected with sterile paper points (STER-I-CELL Paper Points, Size M; Coltene, Whaledent, Cuyahoga Falls, OH, USA) that were inserted into the gingival sulcus for 30 seconds. Plaque samples were collected from the mesiobuccal surfaces of all six Ramfjord teeth and pooled into a single 1.5 ml sterile microcentrifuge tube. Upon collection, plaque samples were stored immediately at −80°C until processing. Samples visibly contaminated with saliva or blood were excluded from the study.

### GCF Chemokine Profiling

After collection, GCF samples were eluted into 200 μl of sample diluent (Bio-Plex Pro™ Human 40-plex Chemokine Panel, Bio-Rad Laboratories, Hercules, CA, USA) with sterile 0.5% bovine serum albumin [Blocker™ BSA (10X) in PBS; Waltham, MA, Thermo Scientific, USA]. Eluted samples were then continuously rotated for 1 h at 4°C. After rotation, soaked paper strips were placed into a basket and microcentrifuge apparatus and spun at 13,000 rpm for 1 min at 4°C to isolate the eluted GCF. Isolated GCF samples were stored at −80°C until further analysis.

Chemokine quantifications were performed simultaneously with a 40-plex immunoassay kit (Bio-Plex Pro™ Human 40-plex Chemokine Panel; Bio-Rad Laboratories, Hercules, CA, USA) undiluted and following all manufacturer's protocols. Multiplex data was obtained using a flow cytometry laser detection system (BioPlex 200 reader; Bio-Rad Laboratories, Hercules, CA, USA) and calculated based on the respective standard curve for each chemokine with a five-parameter logistic (5PL) equation (Bio-Plex Manager Software V6; Bio-Rad Laboratories, Hercules, CA, USA). All mediator concentrations are reported in total amounts per sample collected in 30 seconds (pg per 30-s sample).

Myeloperoxidase (MPO), was quantified separately with an ELISA kit (Human Myeloperoxidase ELISA Kit; Abcam, Cambridge, MA, USA), according to the manufacturer's instructions. Data was measured using a microplate reader at 450 nm (VMax microplate reader; Molecular Devices Sunnyvale, CA, USA) and calculated from a five-parameter logistic (5PL) curve (Softmax Pro Software; Molecular Devices Sunnyvale, CA, USA).

### DNA Extraction and Sequencing of Subgingival Plaque

DNA was extracted from subgingival plaque samples using a commercially available kit (QIAamp DNA Microbiome Kit; Qiagen, Germany) following manufacturer's protocols and 16S rRNA libraries were prepared as previously described [19, 20]. Briefly, after DNA extraction, samples were purified and concentrated (the DNA Clean & Concentrator−5 kit; Zymo Research, Orange, CA, USA), quantitated (Quant-iT dsDNA HS Assay Kit; Invitrogen, Carlsbad, CA, USA) (Qubit 2.0; Life Technologies, Carlsbad, CA, USA), and then stored at −20°C until sequencing. Negative controls for sequencing were performed without plaque samples; and positive controls were run with known bacterial cultures.

For 16s rRNA library preps, hypervariable regions V3 and V4 were targeted using primers (forward: 5′-TCGTCGGCAGCGTCAGATGTGTATAAGAGACAGCCTACGGGNGGCWGC AG-3′; reverse: 5′-GTCTCGTGGGCTCGGAGATGTGTATAAGAGACAGGACTACHVGGGTATCTAATCC-3′) designed with specific flow cell adapter sequences following standard manufacturer's protocol to produce an amplicon of ~460 base pairs (bp) [19]. Amplicons were visually verified on a 1% agarose gel; then subsequently purified with magnetic beads (Agencourt AMPure XP beads; Agencourt Bioscience Corporation, Beckman Coulter Inc., Beverly, MA, USA) and indexed (Illumina Nextera Index Kit; Illumina, San Diego, CA, USA). The indexed PCR amplicons were then further purified with magnetic beads (Agencourt AMPure XP beads; Agencourt Bioscience Corporation, Beckman Coulter Inc., Beverly, MA, USA), and the quality and size of the libraries were assessed with a bioanalyzer (Agilent High Sensitivity DNA Kit & the Agilent 2100 bioanalyzer; Agilent). The resulting libraries from the different samples were then normalized (Quant-iT Picogreen dsDNA Assay Kit; Invitrogen, Carlsbad, CA, USA). Normalized libraries were pooled and paired-end sequencing was carried out on a sequencing platform (MiSeq System, Illumina, San Diego, CA, USA) using a 2 × 300 cycle sequencing kit (MiSeq Reagent Kits v3, Illumina, San Diego, CA, USA).

### Total Bacterial Load

Total bacterial load was determined separately with Quantitative real-time PCR (CFX96 Real-time system C1000 Thermocycler; BioRad Laboratories, Hercules, CA, USA) using a standard curve of serially diluted *Fusobacterium nucleatum* ATCC 10953 genomic DNA (10^8^ to 10^1^ 16s gene copies) with a forward 5′-TCCTACGGGAGGCAGCAGT-3′ and reverse primer 5′-GGACTACCAGGGTATCTAATCCTGTT-3′ set, and TaqMan probe (6-FAM)-5′-CGTATTACCGCGGCTGCTGGCAC- 3′-(TAMRA), (Sigma Aldrich, St Louis, MO, USA) [21]. Negative controls were run with nuclease-free water.

### Sequence Analyses

Analysis of merged 300 bp paired-end reads (average length 450 bp) was performed using Quantitative Insights into Microbial Ecology QIIME2 [22] and Divisive Amplicon Denoising Algorithm 2 (DADA2) [23, 24] as described previously [19, 20]. Taxonomic assignment was performed with the Human Oral Microbiome Database (HOMD 16S rRNA RefSeq V15.1) and a phylogenetic tree was constructed using FastTree [25]. Unrarefied data was used for the downstream analysis. Sequencing data was integrated into a single object using the “phyloseq” R package [26] and all subsequent data analysis and plots were produced in RStudio [27].

Alpha diversity, diversity within samples, was calculated using both richness and evenness metrics by functions estimate_richness() in the “phyloseq” R packages [26]. The community richness was measured by observed species in the sample. The total community diversity (richness and evenness) was measured by Simpson's inverse diversity index [28], and Shannon index [29].

Beta diversity, which evaluates the diversity between samples, was determined using phylogenetic-based Unifrac distances and Bray-Curtis dissimilarity matrix [30, 31]. Beta diversity metrics were calculated with the ordinate() function and were visualized by non-metric multidimensional scaling (NMDS) plots using the plot_oridination() in “phyloseq” R package. The core microbiome was calculated using core() function in “microbiome” package [32].

### Statistical Analyses and Correlations

All statistical analyses were performed using R software version 4.0.4 and RStudio version 1.4.1106 [27, 33]. Clinical and chemokine data were averaged for each subject. Samples with undetectable chemokines were considered zero for the calculations. The correlation between chemokines and neutrophil numbers (MPO) were assessed using the Spearman rank order tests and multiple comparisons were adjusted with the false discovery rate (FDR) method [34]. Principal component analysis (PCA) was performed to examine variation in the chemokine data and identify clusters. Hierarchical clustering of chemokines profiles and microbial communities based on species relative abundances were performed with the hclust() in R using Euclidean distances with Ward's linkage. Heatmaps were created *via* the “clustvis” package in R [35]. The optimal number of clusters was determined using the Silhouette method [36]. The correlation between microbes and chemokine were computed by the Mantel test [37]. Differences in relative abundances of species were determined with LEfSe [38], using an alpha value of 0.01 for the Kruskal–Wallis test and a threshold of 3.5 for logarithmic linear discriminant analysis scores.

## Results

### Clinical Parameters for Study Participants

A total of 20 subjects were enrolled for this study: 12 females (60%) and 8 males (40%); ages ranging between 12 and 17 years, with a mean age of 14.55 ± 1.67 years. All subjects were clinically evaluated and determined to be in good gingival health: no attachment loss, absence of bleeding on probing, probing depths ≤ 3.0 mm, and a gingival index score equal to zero at the time of the study. Overall, the subjects had a mean visible plaque index (VPI) score of 7.78 ± 15.44%, a mean probing depth (PD) of 1.85 ± 0.20 mm, and gingival crevicular fluid (GCF) mean volume of 0.41 ± 0.14 μl per sample for each participant.

### Inter-individual Variability in GCF Chemokines and Neutrophil Profiles in Health

Of the 40 cytokines and chemokines (Table 1) assayed, EOTAXIN-2/CCL24, an eosinophil chemotactic protein, was undetected in all samples and hence excluded from the analysis. In a similar manner, I-309/CCL1, MCP-3/CCL7, IL-4, TARC/CCL17, IL-4, EOTAXIN-3/CCL26, and GM-CSF were only detected in 55–80% of samples, while the rest were detected in more than 90% of the samples. Healthy subjects showed significant inter-individual variability in the levels of cytokines and chemokines (Figure 1A). The levels of mediators were categorized into high (>100 pg per 30-s sample), intermediate (100-10 pg per 30-s sample), and low (<10 pg per 30-s sample) expression within samples.

**Table 1:** Summary of chemokines analyzed from healthy GCF expressed in pg per 30-s sample^*^.

**Chemokine**	**Mean ± SD**	**Min**.	**Max**.
6CKINE/CCL21	55.3 ± 59.94	10.56	251.11
BCA-1/CXCL13	0.86 ± 1.03	0.09	3.64
CTACK/CCL27	0.45 ± 0.28	0.13	1.2
ENA-78/CXCL5	137.76 ± 76.02	0	287.12
EOTAXIN-3/CCL26	1.12 ± 1.19	0	4.63
EOTAXIN/CCL11	0.88 ± 0.38	0.34	1.89
FRACTALKINE/CX3CL1	3.87 ± 3.02	1.3	12.66
GCP-2/CXCL6	9.86 ± 9.5	1.07	38.14
GM-CSF	0.67 ± 0.76	0	2.17
Gro-α/CXCL1	160.42 ± 94.21	9.67	289.83
Gro-β/CXCL2	11.64 ± 9.15	0	34.13
I-309/CCL1	2.13 ± 1.85	0	6.54
I-TAC/CXCL11	0.46 ± 0.59	0.04	1.95
IFN-γ	0.92 ± 0.54	0.3	2.65
IL-10	0.69 ± 0.32	0.13	1.31
IL-16	100.09 ± 66.73	8.89	236.24
IL-1β	51.39 ± 37.23	7.02	135.58
IL-2	0.17 ± 0.1	0.03	0.44
IL-4	0.25 ± 0.21	0	0.75
IL-6	3.37 ± 8.47	0.16	38.92
IL-8/CXCL8	170.98 ± 176.96	12.22	832.26
IP-10/CXCL10	18.69 ± 36.09	0.18	127.78
MCP-1/CCL2	0.82 ± 1.11	0.1	5.05
MCP-2/CCL8	0.18 ± 0.32	0.02	1.45
MCP-3/CCL7	2.76 ± 2.9	0	11.01
MCP-4/CCL13	2.23 ± 1.34	0.19	4.2
MDC/CCL22	0.81 ± 0.58	0.16	2.71
MIF	2683.54 ± 985.82	1202.2	5028.19
MIG/CXCL9	81.25 ± 159.1	2.33	679.05
MIP-1α/CCL3	2.92 ± 3.49	0.17	15.21
MIP-1δ/CCL15	3.42 ± 4.57	0.43	21.29
MIP-3α/CCL20	0.96 ± 1.78	0.09	7.86
MIP-3β/CCL19	4.38 ± 3.27	0.31	12.41
MPIF-1/CCL23	0.49 ± 0.3	0.07	1.23
SCYB16/CXCL16	1.32 ± 1.76	0.11	7.55
SDF-1α + β/CXCL12	4.42 ± 2.02	1.54	8.7
TARC/CCL17	0.74 ± 0.68	0	2.33
TECK/CCL25	43.07 ± 16.71	16.87	80.61
TNF-α	1.76 ± 1.79	0.46	8.69

* *All mediator concentrations are reported in total amounts per sample collected in 30 s (pg per 30-s sample)*.

**Figure 1:** Healthy subjects showed inter-individual variability in GCF chemokine and neutrophil profiles. **(A)** Total amount of chemokines (pg per 30-s sample) in GCF among study participants. MIF was found to be the most abundant chemokine (60–90%) in healthy GCF. **(B)** Myeloperoxidase (MPO), an indirect measure for neutrophils, is highly variable between subjects. **(C)** A Spearman correlogram between MPO and key neutrophil chemokines. Correlation coefficients are expressed by color scale from red (negative correlation) to blue (positive correlation). (*p < 0.05; **p < 0.01; ***p < 0.001).

Highly expressed mediators include: macrophage inhibitory factor (MIF), a neutrophil chemokine, which was the most abundant chemokine in all the samples examined, with a mean value 2683.54 ± 985.82 pg per 30-s sample (Figure 1A). MIF was followed by IL-8/CXCL8, Gro-α/CXCL1, ENA-78/CXCL5, also major neutrophil chemokines, with mean values 170.98 ± 176.96, 160.42 ± 94.21, and 137.76 ± 76.02 pg per 30-s sample, respectively. Intermediately expressed mediators included IL-16 (100.09 ± 66.73 pg per 30-s sample), MIG/CXCL9 (81.25 ± 159.1 pg per 30-s sample), 6CKINE/CCL21 (55.3 ± 59.94 pg per 30-s sample), IL-1β (51.39 ± 37.23 pg per 30-s sample), TECK/CCL25 (43.07 ± 16.71 pg per 30-s sample), IP-10/CXCL10 (18.69 ± 36.09 pg per 30-s sample), and Gro-β/CXCL2 (11.64 ± 9.15 pg per 30-s sample). Low level chemokines included inflammatory mediators, such as GCP-2/CXCL6, IL-6, TNF-α, and IFN-γ with mean values of 9.86 ± 9.5, 3.37 ± 8.47, 1.76 ± 1.79, and 0.92 ± 0.54 pg per 30-s sample, respectively. Interestingly, significant variability was observed in myeloperoxidase (MPO), an indirect measure for neutrophils, within the GCF of healthy individuals with a mean value of 163.16 ± 92.21 ng per 30-s sample ranging from 46.25 to 419.39 ng per 30-s sample (Figure 1B) [39].

A Spearman's rank-order correlation test was performed to identify the relationships between six commonly studied neutrophil chemoattractants and neutrophil concentrations. MIF, GCP-2/CXCL6, and IL-8/CXCL8 showed a significant correlation with the concentration of neutrophils, with the highest correlation between MPO and IL-8/CXCL8 (*r* = 0.54, *P* = 0.14) (Figure 1C). Moreover, an even stronger correlation was observed between IL-8/CXCL8 and ENA-78/CXCL5 (*r* = 0.94, *P* < 0.001).

### GCF Chemokine Phenotypes in Health Separate Into High or Low Expression Groups

To further explore the variability within chemokine profiles between individuals, hierarchical clustering analysis was performed. Clustering analysis generated two groups with different intensities of chemokine pattering: a high and low expression group (Figure 2A). The high expression group included nine participants and was associated with an overall higher chemokine expression. While in contrast, the low expression group, represented by 11 participants, showed an overall lower chemokine expression. Key differences between the groups were within neutrophil chemoattractants such as MIF, IL-8/CXCL8, Gro-α/CXCL1, and ENA-78/CXCL5, in addition to other proinflammatory cytokines such as IL-1β, TNF-α, and IFN-γ. Principal component analysis (PCA) was used to visualize the chemokine data (Figure 2B), where each point represents the chemokine profile of each participant. Individuals with similar chemokine profiles formed two distinct groups, corresponding to the hierarchical groups identified based on chemokine expression intensities. The first principal component (PC1) explained 88.38% of the variation of the data and the second principal component (PC2) explained 11.62%. Thus, this data further demonstrates the wide variability of GCF chemokine expression that is possible to maintain health.

**Figure 2:** GCF chemokines phenotypes in health separate into high or low expression groups. **(A)** A heat map depicting the hierarchical clustering analysis on the 40 chemokines expressions, which generated two groups: high (red) and low (blue). Columns correspond to each of the 20 participants; and rows correspond to each chemokine. Chemokine expression is on a scale of −1 (low; orange) to 4 (high; red). **(B)** A principal component analysis of the chemokines profiles confirmed two distinct groups: high (red) and low (blue). Each point represents a participant.

### Inter-individual Variability of Subgingival Bacterial Communities in Health

The oral microbiome has been shown to play an influential role in host chemokine expression [2, 40]. Therefore, we examined the total bacterial load and subgingival microbial profile of these healthy subjects. 16S rRNA real-time PCR analysis of subgingival plaque samples revealed that the average microbial load was ~10^5^ mean copy numbers, ranging from a low of 10^3.5^ and a high of 10^6^ copy numbers (Figure 3A). Sequencing of the V3-V4 bacterial 16S rRNA gene resulted in a total of 6,736 identified amplicon sequence variants (ASVs) in 20 samples with a total of 863,833 reads, averaging 43,191.65 reads per sample (max = 142,220; min = 1,414; median = 3,3851 reads per sample); and were represented by a total of 10 phyla, 23 classes, 37 orders, 121 genera, and 441 species (Figure 3B). Five phyla were predominant in all subjects: Firmicutes (37.9%), Proteobacteria (19.6%), Bacteroidetes (16.3%), Fusobacteria (12.3%), and Actinobacteria (11.3%). Conversely, Saccharibacteria_(TM7), Spirochaetes, Gracilibacteria_(GN02), Absconditabacteria_(SR1) and Synergistetes were found in low relative abundances in the study participants. The top ten genera identified in all samples were: *Streptococcus, Haemophilus, Fusobacterium, Prevotella, Veillonella, Actinomyces, Porphyromonas, Neisseria, Leptotrichia*, and *Corynebacterium*, representing 75% of the plaque microbiome. The six most abundant species were: *Streptococcus tigurinus* (13.3%), *Streptococcus parasanguinis* (6.3%), *Haemophilus parainfluenzae* (5.3%), *Veillonella dispar* (3.2%), *Haemophilus influenzae* (2.9%), and *Fusobacterium nucleatum* subsp. *animalis* (2.7%). Other low abundance, but more familiar oral bacteria include the genus the Saccharibacteria_(TM7)_[G-1] (2%); and the following species: *Porphyromonas gingivalis* (2.0%), *Streptococcus sanguinis* (1.5%), *Prevotella nigrescens* (1.3%), *Veillonella parvula* (1%), *Prevotella oris* (0.8%), and *Streptococcus mutans* (0.6%).

**Figure 3:** Healthy subjects showed inter-individual variability of subgingival bacterial communities. **(A)** Total bacterial load within subgingival plaque samples across subjects based on 16S qPCR analysis. **(B)** Bar plot of relative taxonomic abundances represented the phylum level across study participants. Five phyla were predominant in all subjects: Firmicutes, Proteobacteria, Bacteroidetes, Fusobacteria, and Actinobacteria. **(C)** Alpha diversity measures using observed species, Shannon index, and Inverse Simpson. Diversity indices show inter-individual variability among study subjects. **(D)** Non-metric multidimensional scaling (NMDS) plots of subgingival samples according to bacterial composition were performed with Bray-Curtis dissimilarity and Unweighted Unifrac distance matrix. Two distinct groups are evident based on the microbial profile. Each point on the graph represents one subject. Each color represents one cluster; A in red and B in blue.

Alpha diversity measurements, which measures differences within samples, showed high variability in the degrees of species richness (observed number of species) within samples (Figure 3C) ranging from 43 to 271 species which averages out to 152.95 observed species per sample. Shannon and Inverse Simpson Indices are common measures of alpha diversity that scores community diversity; a higher score equates to higher diversity. Their respective mean scores were 3.5 and 17.

The microbial community membership and structures were further investigated by beta diversity analyses, which measures differences between samples, using Bray-Curtis and UniFrac distance matrices. Non-metric multidimensional scaling (NMDS) plots of the beta diversity analysis showed separation of the study participants' bacterial communities into two distinct clusters (Figure 3D), meaning that subjects clustered within a group had a more similar microbial composition within other individuals within the same group as opposed to individuals within the other group.

### Low Association Between Sub Gingival Microbiome and GCF Chemokine Expression in Health

Since beta diversity analysis of the microbial data distinguished two separate groups, similar to the chemokine analysis, we examined the possible influence of the oral microbial composition for separation observed within the participant chemokine profiles. The difference in the microbial communities between study subjects was investigated by a hierarchical clustering and differential abundance analysis using species level data.

Interestingly our microbiome analysis revealed two groups (cluster A and cluster B) that were distinct and different from the two chemokine groups identified earlier (Figure 4A). Cluster A was dominated by Firmicutes and Proteobacteria, while cluster B was dominated by Fusobacteria, Bacteroidetes, and Actinobacteria. Moreover, LEfSE analysis identified the key species driving this division (Figure 4B). Cluster A was found to be associated with a mixture of both health- and disease-associated species, such as *Porphyromonas gingivalis*, while in contrast, cluster B was predominated by mostly health-associated bacteria, such as *Rothia dentocariosa*, which is more similar to what has been previously reported in studies investigating oral health [41, 42]. This data suggests that gingival health, defined by clinical parameters, can be achieved by a myriad combination of community compositions and chemokine expressions.

**Figure 4:** Low association between subgingival microbiome and GCF chemokine expression in health. **(A)** Z-score heat map depicting the hierarchical clustering of relative species abundance within subgingival microbial communities. Clustering analysis based on the microbial profile generated two clusters similar to, but different from the chemokine groups; A (red) and B (blue). Each row corresponds to species and each column represents the study subject. Species abundance is on a scale of −1 (low; orange) to 4 (high; red). Color bars in the right depict annotation according to chemokine profile groups and microbiome profile clusters (columns) and phylum (rows). **(B)** Differentially abundant taxa based on LEfSe analysis within the two microbiome clusters (Cluster A, Red and Cluster B, Green). Bars represent linear discriminant analysis scores (LDA) and can be interpreted as the degree of difference in relative abundance.

## Discussion

Chemokines are produced by a variety of cells in the periodontium and play a significant role in the maintenance of oral homeostasis by selective recruitment and activation of key host protective immune cells. Imbalances within these networks have been associated with periodontal disease [42, 43]. In addition, the microbiome has also been shown to be a contributing factor through modulation of host inflammatory responses [2, 10, 44]. Therefore, it is not surprising that much of what is known about oral health is through direct comparisons to either gingivitis or periodontitis. Here, the focus of this cross-sectional study was to examine the chemokine and subgingival microbial profiles of periodontal health.

Our results showed significant inter-individual variability in the number of neutrophils and expression of chemokines during health. Interestingly, we identified two unique chemokine expression patterns that were distinct from clusters identified within the microbial profiles. We suggest that this lack of concordance may be a reflection of the unique combinations between the microbial composition and individualized host response since it well-accepted that chemokine production can be influenced by the microbial composition, environmental factors, and host genetics [7, 11, 45]. Therefore, it is possible that the variation in the chemokine expression levels in health may be useful clues for an individual's susceptibility to disease. For example, several cytokines and chemokines known to be involved in the etiology of periodontal disease were also detected in clinically healthy GCF, such as TNF-α and IL-1β [46, 47]. Furthermore, known disease-associated species including *Treponema denticola, Tannerella forsythia*, and *Porphyromonas gingivalis* were similarly detected in the plaque samples from healthy individuals, but with a low abundance and at a lower frequency [41, 42, 48]. Since periodontitis is associated with a shift in species predominance of subgingival microbial communities rather than as the result of new species colonization, community dysbiosis and associated imbalances in the host inflammatory mediators may lead to a higher susceptibility for a destructive immune response and periodontal tissue destruction [1]. Moreover, a recent study by Bao et al. analyzed correlations between the healthy periodontal tissue proteome and its associated intra-tissue microbiome [49]. In their study, they identified the presence of *Streptococcus vestibularis* and *Veillonella dispar*, which are less invasive oral species, within the layers of healthy gingival tissues without signs of inflammation [49]. Therefore, it is possible that low abundance of more invasive species within some healthy subjects can increase their risk for intra-tissue colonization by normally non-invasive species that can then, have further influences on the maintenance of health.

One major finding of this study is that macrophage migration inhibitory factor (MIF), a key regulatory cytokine of the innate immune system, was the most abundant in all samples examined. MIF levels in healthy GCF showed a significant positive correlation with neutrophil numbers as measured by MPO. Moreover, MIF has been reported to be expressed across the entire human gingival epithelium which is in stark contrast to the human skin, where MIF expression is highly localized to the basal layer [50]. High MIF expression levels in the GCF may be explained by the continuous exposed nature of the gingiva to external stimuli that may induce constitutive expression of MIF by epithelial cells. Therefore, MIF may have an important role in gingival health; however, further studies are required to elucidate its role within gingival homeostasis.

Neutrophil migration into the periodontal tissue is essential for maintaining homeostasis. Three major neutrophil chemokines IL-8/CXCL8, Gro-α/CXCL1, and ENA-78/CXCL5 were among the most abundant chemokines detected in the GCF samples, once again reiterating the important role of neutrophils in maintaining periodontal health. IL-8/CXCL8 is secreted by different gingival cells but the highest expression is preferentially located to the junctional epithelium, which helps in regulating neutrophil influx to periodontal tissues [51]. Similarly, ENA-78/CXCL5, Gro-α/CXCL1, and GCP-2/CXCL6 are involved in neutrophil chemotaxis and activation [52]. Correlation analyses showed that IL-8/CXCL8 was highly associated with neutrophil migration as measured with MPO and both, ENA-78/CXCL5 and Gro-α/CXCL1. However, there were no correlations between ENA-78/CXCL5, Gro-α/CXCL1, and neutrophil numbers. The lack of parallel relationships between these chemokines with neutrophil numbers indicates a complex network orchestrating neutrophil migration and activation during health. Consistent with the variability within chemokine expressions, there was also significant variability in the MPO. The significant correlations between the number of neutrophils (MPO) and neutrophil chemokines IL-8/CXCL8, MIF, and GCP-2/CXCL6, reveal all three of these host mediators significantly contribute to healthy neutrophil migration.

Assessing the expression patterns of a broad range of cytokines and chemokines in health will facilitate our understanding of their role in periodontal pathogenesis. Pro-inflammatory cytokines, IL-1β, IL-6, TNF-α, and IFN-γ, have a major role in the pathogenesis of periodontal disease and were also detected in healthy GCF samples. Since healthy gingival tissue is under constant inflammatory surveillance by neutrophils, this may partially explain the presence of proinflammatory cytokines in healthy GCF [1, 53, 54]. It is of note that anti-inflammatory cytokines IL-4 and IL-10 were also detected in the GCF, emphasizing the importance of the balance between pro-inflammatory and anti-inflammatory cytokines in the healthy periodontium.

In a similar manner to chemokine profiles, there was high variability in the subgingival microbiome profiles between healthy subjects. The uniqueness of the microbial community associated with health has been described where taxa dominating each subject community are highly personalized [55]. The subgingival microbial community was dominated by five phyla; Firmicutes, Proteobacteria, Bacteroidetes, Fusobacteria, and Actinobacteria. Firmicutes (37.9%) was the most predominant phylum in the healthy subgingival plaque in accordance with previous reports [55, 56]. Within the phylum Firmicutes, *Streptococcus tigurinus* (13.3%) and *Streptococcus parasanguinis* (6.3%) were the most abundant taxa among the healthy subgingival plaque as was described previously [42]. Proteobacteria was the second among the most predominant phyla in the healthy subgingival plaque, in contrast with Griffen et al. and Park et al. where Proteobacteria was found to be the most prevalent phylum [41, 57]. These discrepancies between studies could be the result of differences in the target population in addition to differences in the microbial collection and analysis methods. In addition, this study showed a broad range of taxa among healthy individuals. However, a few species were shared by the majority of participants, which included *Streptococcus sanguinis, Streptococcus tigurinus, Streptococcus cristatus, Streptococcus lactarius, Neisseria mucosa*, in addition to *Haemophilus parainfluenzae* and represent the cores species identified within these study participants. Similar results have been described by other reports [41, 42].

Inter-subject variation in the subgingival microbial community was evaluated in the adolescent's healthy population. The study identified two types of microbial communities based on hierarchical clustering techniques, cluster (A) and cluster (B) (Figure 4A). The microbial compositions of the two clusters were different; which was evident by the complete separation of the different clusters microbiome based on beta diversity analysis (Figure 3D). Cluster (B) was dominated by health-associated species whereas cluster (A) was inhabited by health-associated and periodontitis-associated species such as *Porphyromonas gingivalis*. Interestingly, the alpha diversity (within sample diversity) indexes were also variable between the individuals in the different clusters, alpha diversity scores associated with individuals in cluster (A) were noticeably lower, however, higher subgingival bacterial loads were observed (Figure 3A). In agreement, two subgingival community clusters in health were identified in a previous report; one cluster was characterized by higher abundance of the periodontitis-associated genera Porphyromonas and Treponema [58]. Additionally, the two groups identified based on the chemokine expression patterns did not share common microbiome profiles (Figure 4A). This could be attributed to the cross-sectional nature of the study and the dynamic nature of the host response and microbiome. Thus, assessment of the microbial community composition and host response variation between individuals is crucial in understanding the microbiome and host factors involvement with disease risks.

Few studies have investigated the influence of the microbial community composition on the host response in the healthy periodontal tissue. The Mantel test revealed no significant correlation between combined chemokines and microbiome profiles in this study. Interestingly, further analyses found significant correlations between the core species and neutrophil chemokines. However, it is important to note that this study has several potential limitations, which includes the cross-sectional design of this study and the small sample size. Hence, keep in mind that this brief snap-shot in time may have only captured a transient moment within the larger regulatory context and may not affect overall health or disease. Moreover, this study did not consider variations within individual diets, nor account for differences within natural circadian rhythms. Therefore, a deeper more robust analysis may produce a more concrete level of correlation between the microbiome and chemokine data. Lastly, pooling of subgingival microbial samples may have resulted in the loss of site-specific data [59]. Therefore, evaluating changes within larger chemokine and microbiome profiles during a longitudinal trial from health to disease would be ideal. Yet, despite these limitations, the results of this study revealed that the inter-individual variability with the number of neutrophils, chemokine expression, and microbial profile during health, which has been previously uncharacterized, is a complexity of healthy oral homeostasis.

## Data Availability Statement

The datasets generated for this study can be found in online repositories. The name of the repository and accession number can be found below: NCBI Short Read Archive (SRA) under BioProject PRJNA728740 (https://www.ncbi.nlm.nih.gov/Traces/study/?acc=PRJNA728740&o=acc_s%3Aa).

## Ethics Statement

The studies involving human participants were reviewed and approved by The University of Washington's Human Subjects Review Committee (HSD#46857). Written informed consent to participate in this study was provided by the participants' legal guardian/next of kin.

## Author Contributions

SB, JM, and RD designed the study. SB contributed to the collection of samples and clinical data. SB, SJ, and AC performed laboratory experiments. SB, GK, and JM conducted statistical and bioinformatics analyses. SB, AC, and RD wrote the manuscript. All authors contributed to the article and approved the submitted version.

## Conflict of Interest

The authors declare that the research was conducted in the absence of any commercial or financial relationships that could be construed as a potential conflict of interest.
